This article has been retracted.

# MicroRNA-595 sensitizes ovarian cancer cells to cisplatin by targeting ABCB1

**DOI:** 10.18632/oncotarget.13526

**Published:** 2016-11-23

**Authors:** Songyu Tian, Mingyue Zhang, Xiuwei Chen, Yunduo Liu, Ge Lou

**Affiliations:** ^1^ Department of Gynecology Oncology, Cancer Hospital of Harbin Medical University, Harin, 150081, Heilongjiang, China; ^2^ Department of Anaesthesiology, Cancer Hospital of Harbin Medical University, Harin, 150081, Heilongjiang, China

**Keywords:** ovarian cancer, microRNAs, miR-595, ABCB1

## Abstract

Ovarian cancer is among the leading cause of cancer-related deaths in females. In this study, we demonstrated that miR-595 expression was downregulated in the ovarian cancer tissues and cell lines. miR-595 expression was lower in the lymph node metastases tissues than in the primary ovarian cancer tissues and normal tissues. Furthermore, miR-595 overexpression suppressed the ovarian cancer cell proliferation, colony formation and invasion and promoted the sensitivity of ovarian cancer cell to cisplatin. We identified ABCB1 as a direct target gene of miR-595 in the ovarian cancer cell. ABCB1 expression was upregulated in the ovarian cancer tissues and cell lines. Morevoer, the expression level of ABCB1 was inversely correlated with miR-595 in the ovarian cancer tissues. In addition, overexpression of ABCB1 decreased the miR-595-overexpressing HO8910PM and SKOV-3 cell sensitivity to cisplatin. Ectopic expression of ABCB1 promoted the miR-595-overexpressing HO8910PM and SKOV-3 cell proliferation, colony formation and invasion. These data suggested that miR-595 acted a tumor suppressor role in ovarian cancer development and increased the sensitivity of ovarian cancer to cisplatin.

## INTRODUCTION

Epithelial ovarian cancer accounts for approaximately 90% of ovarian cancers and comprises of many different subgroups according to their histological origins, including serous, mucinous, endometrioid, undifferentiated, clear celland Brenner carcinomas [1–4]. Diagnosis of early-stage ovarian cancer is challenging since it manifests few symptoms [5, 6]. Although many diagnostic approaches are developed, most patients are not diagnosed until it is at an advanced stage [7–10]. The 5-year survival rate of advanced ovarian cancer is only 20–25% [2, 11–13]. Therefore, it is urgent to explore sensitive and specific diagostic biomarkers for ovarian cancer to improve patient’s survival.

MicroRNAs (miRNAs) are a group of endogenous, 18–25 nucleotides long, non-coding RNAs that inhibit gene expression through binding to the 3′UTR of their target mRNAs and induce mRNA cleavage and inhibit the protein translation [14–18]. miRNAs are involved in a lot of important cell biological processes such as cell development, growth, apoptosis, differentiation, migration and invasion [19–22]. Growing evidences have demonstrated that dysregulation of miRNAs is found in many tumors and plays critical roles in the development, initiation and metastasis of tumors [18, 23–25]. Recently, miRNA have been found to be involved in the drug resistance in many cancers [20, 26, 27].

Recently, several reports have demonstrated that miR-595 plays crucial roles in the progression of various tumors [28–30]. For example, Hao et al [28]. demonstrated that the miR-595 expression was upregulated in the glioblastoma cells and tissues. Overexpression of miR-595 increased the glioblastoma cell proliferation and colony formation through inhibiting SOX7. Chen et al [31]. demonstrated that miR-595 regulated the neuroblastoma cells SH-SY5Y autophagy by repressing ULK1 expression. However, the underlying mechanism of miR-595 in ovarian cancer was still not well elucidated. In this study, we demonstrated that miR-595 expression was downregulated in the ovarian cancer tissues and cell lines. miR-595 overexpression suppressed the ovarian cancer cell proliferation, colony formation and invasion and promoted the sensitivity of ovarian cancer cell to cisplatin. We identified ABCB1 as a direct target gene of miR-595 in the ovarian cancer cell.

## RESULTS

### miR-595 expression increased the sensitivity of HO8910PM cells to cisplatin

We firstly measured the expression of miR-595 in 5 ovarian cancer cell lines (HG-SOC, HO8910, SKOV-3, HO8910PM and ES2) and immortalized normal fallopian tube epithelial cell line (FTE187). Our data suggested that miR-595 expression was lower in the ovarian cancer cell lines than in the FTE187 cell (Figure 1A). The expression of miR-595 was upregulated in the HO8910PM cell (Figure 1B) and SKOV-3 (Figure 1D) after threated with miR-595 mimic. The HO8910PM cell and SKOV-3 cell response to cisplatin increased after treated with the miR-595 mimic compared with control-transfected cells (Figure 1C and 1E).

**Figure 1:** miR-595 increased the sensitivity of HO8910PM cells to cisplatin (**A**) The miR-595 expression in the 5 ovarian cancer cell lines (HG-SOC, HO8910, SKOV-3, HO8910PM and ES2) and immortalized normal fallopian tube epithelial cell line (FTE187) was determined by qRT-PCR. (**B**) The expression of miR-595 in the HO8910PM cell after treated with miR-595 mimic was measured using qRT-PCR. (**C**) The HO8910PM cell response to cisplatin was increased after treated with the miR-595 mimic. (**D**) The expression of miR-595 in the SKOV-3 cell after treated with miR-595 mimic was measured using qRT-PCR. (**E**) The SKOV-3 cell response to cisplatin was increased after treated with the miR-595 mimic. *p < 0.05, **p < 0.01 and ***p < 0.001.

### miR-595 expression was downregulated in ovarian cancer tissues

miR-595 expression was downregulated in the ovarian cancer tissues compared to the matched normal ovarian tissues (Figure 2A). miR-595 expression was downregulated in 29 ovarian cancer tissues (29/35; 74.2%) compared to the adjacent tissues (Figure 2B). miR-595 expression was lower in the lymph node metastases tissues compared to the primary ovarian cancer tissues and the normal tissues (Figure 2C).

**Figure 2:** miR-595 was downregulated in ovarian cancer tissues (**A**) The expression of miR-595 in the ovarian cancer tissues was determined by qRT-PCR. (**B**) Among these, the miR-595 expression was downregulated in the 29 ovarian cancer tissues (29/35; 74.2%) compared to the adjacent tissues. (**C**) miR-595 expression in the lymph node metastases tissues and the primary ovarian cancer tissues and the normal tissues was measured by qRT-PCR. *p < 0.05 and ***p < 0.001.

### Ecotpic expression of miR-595 inhibited ovarian cancer cell proliferation, colony formation and invasion

Ectopic expression of miR-595 inhibited the HO8910PM and SKOV-3 cell proliferation (Figure 3A and 3D). In line with these, miR-595 overexpression suppressed the expression of ki-67 and PCNA in the HO8910PM cell (Figure 3B and 3C). Overexpression of miR-595 inhibited the expression of ki-67 and PCNA in the SKOV-3 cell (Figure 3E and 3F). Ectopic expression of miR-595 inhibited the HO8910PM and SKOV-3 cell colony formation (Figure 3G and 3H). In addition, overexpression of miR-595 suppressed the HO8910PM and SKOV-3 cell invasion (Figure 3I and 3J).

**Figure 3:** Ecotpic expression of miR-595 inhibited ovarian cancer cell proliferation, colony formation and invasion (**A**) Overexpression of miR-595 suppressed the HO8910PM cell proliferation. (**B**) Ecoptic expression of miR-595 inhibited the ki-67 expression in the HO8910PM cell. (**C**) Overexpression of miR-595 suppressed PCNA expression in the HO8910PM cell. (**D**) Overexpression of miR-595 suppressed the SKOV-3 cell proliferation. (**E**) Overexpression of miR-595 suppressed the ki-67 expression in the SKOV-3 cell. (**F**) Elevated expression of miR-595 decreased the PCNA expression in the SKOV-3 cell. (**G**) Overexpression of miR-595 suppressed the HO8910PM cell colony formation. The relative conoly number was shown in the right. (**H**) Elevated expression of miR-595 decreased the SKOV-3 cell colony formation. The relative conoly number was shown in the right. (**I**) miR-595 overexpression inhibited the HO8910PM cell invasion. The relative invasive cells were shown in the right. (**J**) Elevated expression of miR-595 suppressed the SKOV-3 cell invasion. The relative invasive cells were shown in the right. *p < 0.05, **p < 0.01 and ***p < 0.001.

### ABCB1 was a direct target of miR-595 in the ovarian cancer cell

As predicted by TargetScan, ABCB1 was a potetial target gene of miR-595 (Figure 4A). The effect of miR-595 on ABCB1 mRNA translation into protein was measured by a luciferase reporter assay (Figure 4B). miR-595 overexpression inhibited the luciferase activity of wild-type reporter but not the mutant ABCB1 3′UTR reporter (Figure 4B). Ectopic expression of miR-595 inhibited ABCB1 mRNA and protein expression in HO8910PM cells (Figure 4C and 4D).

**Figure 4:** ABCB1 was a direct target of miR-595 in the ovarian cancer cell (**A**) ABCB1 was a potetial target gene of miR-595 by using TargetScan system. (**B**) The effect of miR-595 on ABCB1 mRNA translation into protein was measured by a luciferase reporter assay. (**C**) Ectopic expression of miR-595 inhibited ABCB1 mRNA expression in HO8910PM cells. (**D**) Ecotopic miR-595 expression inhibited the ABCB1 protein expression in the HO8910PM cells. ***p < 0.001.

### The expression of ABCB1 was upregulated in the ovarian cancer tissues

Compared with matched non-tumor tissues, ABCB1 was higher in the ovarian cancer tissues (Figure 5A). Among these, the ABCB1 expression was upregulated in the 25 ovarian cancer tissues (25/35; 71.4%) compared to the adjacent tissues (Figure 5B). ABCB1 expression was higher in the ovarian cancer cell lines compared to in the FTE187 cell (Figure 5C). Interestingly, among pairs of ovarian cancer tissues and non-tumor tissues, ABCB1 expression was inversely correlated with miR-595 expression (Figure 5D).

**Figure 5:** The expression of ABCB1 was upregulated in the ovarian cancer tissues (**A**) ABCB1 expression was upregulated in the ovarian cancer tissues compared to matched non-tumor tissues. (**B**) Among these, the ABCB1 expression was upregulated in the 25 ovarian cancer tissues (25/35; 71.4%) compared to the adjacent tissues. (**C**) The expression of ABCB1 was determined in the ovarian cancer cell lines and FTE187 cell. (**D**) The expression of ABCB1 was inversely associated with the miR-595 expression in the ovarian cancer tissues.

### miR-595 promoted the sensitivity of HO8910PM cells to cisplatin and inhibited ovarian cancer cell proliferation, colony formation and invasion through targeting ABCB1

The expression of ABCB1 was upregulated in the HO8910PM cell after treated with the ABCB1 vector (Figure 6A and 6B). The responses of HO8910PM and SKOV-3 cell to cisplatin were decreased after transfected with the ABCB1 vector compared with the control vector (Figure 6C and 6D). In addition, the responses of miR-595-overexpressing HO8910PM and SKOV-3 cell to cisplatin were also decreased after transfected with the ABCB1 vector compared with the control vector (Figure 6F and 6I). Ecotopic expression of ABCB1 promoted the HO8910PM and SKOV-3 cell proliferation (Figure 6E and 6G). Overexpression of ABCB1 increased miR-595-overexpressing HO8910PM and SKOV-3 cell proliferation (Figure 6H and 6J). Moreover, ectopic expression of ABCB1 promoted the miR-595-overexpressing HO8910PM and SKOV-3 cell colony formation (Figure 6K and 6L). In addition, elevalted expression of ABCB1 increased the miR-595-overexpressing HO8910PM and SKOV-3 cell invasion (Figure 6M and 6N).

**Figure 6:** miR-595 promoted the sensitivity of HO8910PM cells to cisplatin and inhibited ovarian cancer cell proliferation, colony formation and invasion through targeting ABCB1 (**A**) The mRNA expression of ABCB1 was increased in the HO8910PM cell after treated with the ABCB1 vector. (**B**) The protein expression of ABCB1 in the HO8910PM cell was determined by Western blot. (**C**) Overexpression of ABCB1 decreased the HO8910PM cell response to cisplatin. (**D**) Overexpression of ABCB1 decreased the SKOV-3 cell response to cisplatin. (**E**) Overexpression of ABCB1 increased SKOV-3 cell proliferation. (**F**) The responses of miR-595-overexpressing HO8910PM cells to cisplatin were decreased after transfected with the ABCB1 vector. (**G**) Ecotopic expression of ABCB1 promoted the HO8910PM cell proliferation. (**H**) Overexpression of ABCB1 increased miR-595-overexpressing HO8910PM cell proliferation. (**I**) The responses of miR-595-overexpressing SKOV-3 cells to cisplatin were decreased after transfected with the ABCB1 vector. (**J**) Overexpression of ABCB1 increased miR-595-overexpressing SKOV-3 cell proliferation. (**K**) Overexpression of ABCB1 increased the miR-595-overexpressing HO8910PM cells colony formation. The relative conoly number was shown in the right. (**L**) Overexpression of ABCB1 increased the miR-595-overexpressing SKOV-3 cells colony formation. The relative conoly number was shown in the right. (**M**) Overexpression of ABCB1 increased the miR-595-overexpressing HO8910PM cells invasion. The relative invasive cells were shown in the right. (**N**) Overexpression of ABCB1 increased the miR-595-overexpressing SKOV-3 cells invasion. The relative invasive cells were shown in the right. *p < 0.05, **p < 0.01 and ***p < 0.001.

## DISCUSSION

In this study, we demonstrated that miR-595 expression was downregulated in the ovarian cancer tissues and cell lines. miR-595 expression was lower in the lymph node metastases tissues than in the primary ovarian cancer tissues and the normal tissues. Furthermore, miR-595 overexpression suppressed the ovarian cancer cell proliferation, colony formation and invasion and promoted the sensitivity of ovarian cancer cell to cisplatin. We identified ABCB1 as a direct target gene of miR-595 in the ovarian cancer cell. ABCB1 expression was higher in the ovarian cancer tissues and cell lines. The expression level of ABCB1 was inversely correlated with miR-595 in the ovarian cancer tissues. In addition, overexpression of ABCB1 decreased the miR-595-overexpressing HO8910PM cell sensitivity to cisplatin. Moreover, our data demonstrated that ectopic expression of ABCB1 promoted the miR-595-overexpressing HO8910PM cells proliferation, colony formation and invasion. These data suggested that miR-595 acted a tumor suppressor role in ovarian cancer development and increased the sensitivity of ovarian cancer to cisplatin.

Recently, several reports have demonstrated that miR-595 plays important roles in the development of many tumors [28–30]. For example, Hao et al. [28]. showed that the expression of miR-595 was upregulated in the glioblastoma cells and tissues. Overexpression of miR-595 promoted the glioblastoma cell proliferation and colony formation through targeting SOX7. Another study demonstrated that miR-595 expression was upregulated in the sera of active forms of inflammatory bowel disease patients [32]. Chen et al. [31]. showed that miR-595 regulated the neuroblastoma cells SH-SY5Y autophagy through targeting ULK1. However, the underlying mechanism of miR-595 in ovarian cancer was still not well elucidated. In our study, we firstly determined the expression of miR-595 in the ovarian cancer cell and tissues. Our data showed that miR-595 expression was lower in the ovarian cancer cell lines than in the FTE187 cell. Furthermore, the expression of miR-595 was downregulated in the ovarian cancer tissues compare to their matched normal ovarian tissues. miR-595 expression was lower in the lymph node metastases tissues compared to the primary ovarian cancer tissues and the normal tissues. In addition, overexpression of miR-595 suppressed the ovarian cancer cell proliferation, colony formation and invasion.

Drug resistance is considered to be the major cause to the success of tumor chemotherapy [33–36]. Several studies demonstrated that miRNAs acted an important role in the drug resistance [37–39]. MiRNAs can modulate various genes expression and play critical roles in tumor cell apoptosis, proliferation and cell cycle, lead to different cellular sensitivity or resistance to chemotherapeutic agents [40, 41]. In this study, our data found that ectopic expression of miR-595 promoted the sensitivity of HO8910PM cells to cisplatin. These findings suggested that miR-595 acted sensitizes ovarian cancer cells to cisplatin.

ABCB1 belongs to the ABC transporter family and is located on the chromosome 7 [42, 43]. The ABC family contains about 12 putative drug transporters, such as MRP1 (MDR-associated protein-1, encoded by ABCC1) and MDR1 (encoded by ABCB1) [44, 45]. ABCB1 participates in efflux of drugs from tumor cells [46, 47]. In addition, ABCB1 overexpression is considered to contribute to the drug resistance in various cancers [48]. In our study, we showed that ABCB1 was a direct target gene of miR-595 in ovarian cancer. Ectopic expression of miR-595 inhibited the luciferase activity of the wild-type reporter but not of the mutant ABCB1 reporter, suggesting that miR-595 could directly regulate the ABCB1 expression. Furthermore, miR-595 overexpression suppressed ABCB1 expression in HO8910PM cells. We also investigated that ABCB1 expression was higher in ovarian cancer tissues and cells, and inversely correlated with miR-595 expression in ovarian cancer tissues. MiR-595 suppressed ovarian cancer cell proliferation, colony formation and invasion through targeting ABCB1. Moreover, ABCB1 overexpression decreased the sensitivity of miR-595-overexpressing HO8910PM cells to cisplatin in ovarian cancer. These data suggested that the ability of miR-595 to target ABCB1 may represent a potential mechanism for the post-transcriptional control for ABCB1 expression.

In summary, we showed that miR-595 was downregulated in the ovarian cancer cell and tissues. Ectopic expression of miR-595 suppressed the ovarian cancer cell proliferation, colony formation and invasion and promoted the ovarian cancer cell response to cisplatin through targeting ABCB1. These data suggested that miR-595-ABCB1 was a potential therapeutic target for patients with ovarian cancer.

## MATERIALS AND METHODS

### Tissue samples and cell lines culture and tranfection

Human epithelial ovarian tumor tissues and their matched normal ovarian tissues were obtained from our hospital during surgery. None of these patients were received radiotherapy and chemotherapy before surgery. This study was approved by the Ethics Committee of Cancer Hospital of Harbin Medical University. Five ovarian cancer cell lines (HG-SOC, HO8910, SKOV-3, HO8910PM and ES2) and one immortalized normal fallopian tube epithelial cell line (FTE187) were purchased from the Type Culture Collection (Shanghai, China). The cells were kept in the RPMI-1640 medium contained with fetal serum (Invitrogen, USA). miR-595 mimic and the control scramble miRNA were purchased from Gene Pharma (Shanghai, China). Cell transfection was performed by Lipofectamine 2000 (Invitrogen, USA) following to the instruction.

### Quantitative real-time PCR

Total RNA from the cells or tissues was extracted by using TRIzol reagent (Invitrogen, USA) according to the instructions. cDNA was synthesized with the miRNA-specific primer or oligo(dT) using the Synthesis System for RT-PCR (Invitrogen, USA). Quantitative real-time PCR was done to measure the miR-595 and mRNA expression by using SYBR Green PCR mix (Applied Biosystems, CA, USA) on the ABI 7500 System following to the manufacturer’s instructions. U6 and GAPDH were used as an internal control for miR-595 and mRNA expression respectively.

### Dual luciferase activity assay

Cells were cultured in the 12-well plates and were transfected with pGL3-ABCB1-3′UTR-MUT or pGL3-ABCB1-3′UTR-WT vector and miR-595 mimic or scramble oligonucleotide using Lipofectamine-2000 (Invitrogen, USA) according to the manufacturer’s instructions. After 48 h, luciferase activity was determined using the Dual-Luciferase Reporter System (Promega, USA). Data are shown as the ratios between firefly and Renilla activities.

### Western blot

Total protein was extracted from cell or tissue by using RIPA lysis buffer and the protein concentration was determined using BCA Protein Assay kit. The total protein was separated on 12% SDS-PAGE gels and then transferred to the membrane. The membrane was blocked and then incubated with primary antibodies (ABCB1, Santa Cruz, USA) and GAPDH (Abcam, USA) (each 1:5000). The membrane was probed with horseradish peroxidase-labeled secondary antibody. Signa was visualized using ECL (enhanced chemiluminescence detection system). GAPDH was used as the control.

### Cell proliferation, invasion and colony formation assays

Cell proliferation was evaluated by using CCK-8 (Cell Counting Kit-8) according to the manufacturer’s instructions. Cells were cultured in the 96-well plate and incubated for 24 h, 48 h and 72 h respectively. CCK-8 reagent (10 mL) was put to each well and incubated for 2–3 h. The absorbance value at 450 nm was measured by the microplate reader. For colony formation analysis, cells were plated in the 6-well plates and were incubated for 2 weeks. Colonies were fixed and stained with the crystal violet and counted. The invasive potential of cells was determined by transwell inserts. Cells were cultured in the upper insert coated with the matrigel matrix (BD). FBS (10%) medium was put into the lower chamber. After 48 h, noninvaded cell was removed with the cotton swab and was fixed with methanol, stained with the crystal violet and counted.

### Statistical analysis

Student’s *t-test* or one-way ANOVA was used to measure the statistical significance between groups by using SPSS 17.0 software. *P <* 0.05 was considered significant difference and Data was shown as means ± SD (standard deviation).
